The article "Exploration of the Potential Mechanism of the Common Differentially Expressed Genes in Psoriasis and Atopic Dermatitis" was published in 2022. Journal: Biomed Res Int.

# Exploration of the Potential Mechanism of the Common Differentially Expressed Genes in Psoriasis and Atopic Dermatitis

**DOI:** 10.1155/2022/1177299

**Published:** 2022-05-09

**Authors:** Zhiyu Zhou, Li Meng, Yawen Cai, Wannian Yan, Yun Bai, Jia Chen

**Affiliations:** ^1^Department of Dermatopathology, Shanghai Skin Disease Hospital, Tongji University School of Medicine, Shanghai, China; ^2^Department of Central Laboratory, Shanghai Skin Disease Hospital, Tongji University School of Medicine, Shanghai, China

## Abstract

**Backgrounds:**

Psoriasis and atopic dermatitis are two common chronic inflammatory skin diseases that enormously deteriorate the psycho-physical and socio-economic condition of the patients. Although differential immune responses have been found to operate in the pathomechanisms of atopic dermatitis and psoriasis, the epidermal keratinocytes are the major targets in both diseases, and sometimes, they show similar clinical presentations. The skin barrier, itching, and inflammation are current and future treatment targets for both of them, but the relevant shared mechanisms of the two diseases are far from understood.

**Methods:**

The differential analyses of GSE14905 (psoriasis) and GSE32924 (atopic dermatitis) deposited in GEO database were conducted and obtained their differential expressed genes. Moreover, PPI, functional modules, GO, and KEGG enrichment analyses were used for the further analysis. The mouse models of psoriasis and atopic dermatitis were established, and then, RT-qPCR and Western blotting assay were performed to check the abundant changes of hub genes.

**Results:**

There are 732 differentially expressed genes in psoriasis versus nonlesional skin samples. Besides, 611 differentially expressed genes were identified in atopic dermatitis versus nonlesional skin data sets. Based on these differentially expressed genes, we predicted their joint and individual protein-protein interaction networks and functional modules in both psoriasis and atopic dermatitis. Through the PPI network of genes, we calculated the hub nodes and do the GO and KEGG enrichment analysis of overlapped genes of psoriasis and atopic dermatitis, which suggested there were some terms like “positive regulation of interleukin-12 production,” “centromeric region,” and “TNF signaling pathway.”

**Conclusion:**

We constructed the predicted PPI networks and functional modules related to psoriasis and atopic dermatitis and distinguished the key candidate target genes *CXCL8*, *STAT1*, and *MMP9* in the diagnosis and therapy of similar pathogenesis.

## 1. Introduction

Psoriasis is a chronic inflammatory disease characterized by periodic continuous inflammation and relief, uncontrolled proliferation of keratinocytes, and impaired differentiation of keratinocytes [1–3]. The prevalence in adults ranged from 0.51% to 11.43% and in children from 0% to 1.37% while differ according to regions [4]. It was reported that the prevalence was low in Asian and African populations and high in Caucasian and Scandinavian populations [5, 6]. Inflammation in patients with psoriasis is caused by abnormalities of innate or adaptive immunity system and has obvious inheritance tendency [7–9]. Psoriatic patients are usually categorized into three groups according to the situation such as clinical severity, the percentage of affected body surface area, and patient quality of life and the treatments are different [10]. Mild psoriasis can be treated with topical agents, phototherapy for moderate disease, and systemic agents for severe disease [11–13].

The article "Exploration of the Potential Mechanism of the Common Differentially Expressed Genes in Psoriasis and Atopic Dermatitis" was published in 2022. Journal: Biomed Res Int.

Atopic dermatitis (AD) is a chronic and recurrent inflammation of the skin associated with symptoms such as pruritus, sleep disturbance, depression, and anxiety [14–18]. It was reported that the 1-year prevalence of doctor-diagnosed AD ranged from 1.2% in Asia, to 17.1% in Europe in adults, and 0.96% to 22.6% in children in Asia in the 21 century [19]. There are two competing hypotheses for the occurrence of AD: the “inside-out” hypothesis suggests that physical changes in the epidermal structure drive immune dysregulation, whereas the “outside-in” hypothesis favors the point that aberrant immune activity alters the skin-barrier [20–23]. Because of the complex pathogenesis, treatment used for AD is more complicated than for psoriasis [24]. It is thus desirable to develop well-tolerated medicine for AD patients.

Psoriasis and atopic dermatitis are two common chronic skin diseases [25]. Both are related to the imbalance of Th1/Th2 cells in the immune system and show an antagonistic mechanism, that is, psoriasis is mainly mediated by Th1 cells, while atopic dermatitis is mainly mediated by Th2 cells. Sometimes, atopic dermatitis and psoriasis appear simultaneously in a same patient, which poses a challenge to the doctors. Because of the similar pathogenesis, psoriasis and atopic dermatitis were considered as part of the same disease spectrum [24, 26, 27]. Analyzing psoriasis and atopic dermatitis together may contribute to a deeper understanding of the diseases and improve the therapy. In this study, we analyzed the gene expression pattern by reanalyzing the data of GSE14905 (psoriasis) and GSE32924 (atopic dermatitis) deposited in Gene Expression Omnibus (GEO) database. Differentially expressed genes (DEGs) were identified, and gene function enrichment analysis was performed for psoriasis and atopic dermatitis, respectively. Then, PPI networks and key modules in psoriasis and atopic dermatitis were constructed by using above-mentioned DEGs. Furthermore, the intersection of psoriasis and atopic dermatitis data sets were used to analyze the common characteristics. Finally, the expression levels of several genes were detected and validated by RT-qPCR and Western blot in disease mouse models (Figure 1).

The article "Exploration of the Potential Mechanism of the Common Differentially Expressed Genes in Psoriasis and Atopic Dermatitis" was published in 2022. Journal: Biomed Res Int.

## 2. Materials and Methods

### 2.1. Data Mining of GEO Database

Two sets of databases, GSE14905 (psoriasis) and GSE32924 (atopic dermatitis), were obtained from gene expression omnibus (GEO, http://www.ncbi.nlm.nih.gov/geo/). GSE14905 contains 61 expression data sets of psoriasis samples, including 33 samples of lesional skin and 28 samples of nonlesional skin. GSE32924 contains 25 expression data sets of atopic dermatitis samples, including 13 samples of lesional skin and 12 samples of nonlesional skin.

### 2.2. Data Preprocessing

GSE14905 and GSE32924 data sets were debatched. The limma [28] package was used to normalize the obtained chip expression data by quartile. Then, log2 logarithmic transformation is performed to finally obtain the gene expression matrix of the sample group. R package limma [28] was used to perform the different expression analysis of genes between the psoriasis/atopic-dermatitis samples and the healthy samples using the expression matrix. The screening threshold for significant differences in gene expression was *P* < 0.05 and |log2FC| > 0.585 (i.e., FC > 1.5 or FC < 1/1.5).

### 2.3. PPI Network Prediction

The protein-protein interactions (PPIs) of genes were analyzed by string [29] online tool. The threshold of combined score in protein-protein interactions is 5. From the perspective of obtained biological networks, the topology of PPI relation network was analyzed by Cytoscape through pairs with PPI relationship. Therefore, the important nodes with protein-protein interaction relationships in PPI networks were obtained by the connectivity degree analysis in network statistics [30]. Here, we analyzed the nodes of the PPI network.

### 2.4. Gene Function Enrichment Analysis

Based on the database of Gene Ontology [31] and the database of biochemical pathways KEGG pathway database [32], the candidate genes were conducted functional enrichment by clusterProfiler [33] using the Fisher's exact test.

### 2.5. Stem-Lop RT-qPCR

The primers used in the stem-lop RT-qPCR were synthesized and listed in Table 1. cDNA was generated by reverse transcription using 1 *μ*g RNA as template. Then, stem-loop and U6 RT primers were combined to transcribe the total RNA. RT-qPCR was performed using the SYBR Premix Ex Taq II kit following the manufacturer's protocol, and fluorescence intensity was measured. All experiments were performed 20 times.

The article "Exploration of the Potential Mechanism of the Common Differentially Expressed Genes in Psoriasis and Atopic Dermatitis" was published in 2022. Journal: Biomed Res Int.

### 2.6. Establishment of Animal Model

Thirty 6-8-week-old mice with 18-22 g body weight were divided into normal group, psoriasis model group, and atopic dermatitis model group. After back depilation of mice, the normal group applied Vaseline on the back of mice every day; psoriasis model group and atopic dermatitis model group applied imiquimod cream and oxazolone separately on the back of mice daily for 21days. The mice were sacrificed on the 22nd day of modeling, and the skin lesions on the back were cut for histopathological examination. Gross and pathological morphology of skin lesions were used to determine the incidence of psoriasis and atopic dermatitis.

### 2.7. Western Blot

Proteins were extracted from fresh mouse skin tissue with RIPA lysis buffer (Beyotime Biotechnology). Protein samples (60 *μ*g) were separated by SDS-PAGE electrophoresis and transferred to PVDF membranes (Millipore) at 20 V for 1 h. After blocking with 5% nonfat dry milk in TBS, the protein on the membrane was incubated with primary antibody (appropriate dilution for CXCL8, STAT1, PTPRC, *β*-actin, and MMP9, respectively) at 4°C overnight. The following primary antibodies were used: anti-*β* actin (CST, MA, USA, #4970, 1 : 1000); anti-STAT1 (ab234400, 1: 1000, Abcam), anti-MMP9 antibody (ab76003, Abcam, Cambridge, MA, USA), anti-CXCL8 recombinant antibody (CAT#: TAB-201CL), and anti-CD45 monoclonal antibody (DCABH-1351). After four washes for 5 minutes in TBST, the secondary antibody was incubated in an appropriate dilution for 1 h at room temperature followed by four washes for 5 minutes in TBST. Then, FluorChemE imager (Alpha) was used for visualization, and the expression level of specific protein was normalized to *β*-actin level. This study got the vertebrate animal study approval from Shanghai Dermatology Hospital Clinical Trial Ethics Committee (SSDH-IEC-SG-057-3.1).

### 2.8. Statistical Analysis

Statistical software SPSS 16.0 (SPSS Inc.) was used for data processing, and one-way ANOVA was used for statistical analysis between 3 groups and more than 3 groups. Wilcoxon rank-sum test was used for statistical analysis between 2 groups. When *P* < 0.05, the difference was statistically significant.

## 3. Results

### 3.1. Identification of DEGs in Psoriasis and Atopic Dermatitis

33 expression data sets of psoriasis lesional skin and 28 expression data sets of psoriasis nonlesional skin were available for further analysis. 732 differentially expressed genes were obtained between them with the threshold of fold change (FC) > 1.5 and *P* value < 0.05, and the expression value of DEGs among each sample was shown in Figure 2(a). The correlation of gene expression levels between samples is a crucial measure of the reliability of experiments and samples. Apart from two samples (GSM372333 and GSM372352), the other samples are well classified by using the DEGs. To explore the enrichment pathways, GO and KEGG analyses were performed. The most significantly enriched BP term and KEGG pathway were “T cell activation” and “cytokine-cytokine receptor interaction”, respectively (Figures 2(b) and 2(c)). Furthermore, the GO terms “response to virus,” “response to molecular of bacterial origin,” “defense response to virus,” “cytokine secretion,” and “cornification” were enriched as well.

The article "Exploration of the Potential Mechanism of the Common Differentially Expressed Genes in Psoriasis and Atopic Dermatitis" was published in 2022. Journal: Biomed Res Int.

DEG analysis was also performed for the 13 expression data sets of atopic dermatitis lesional and 12 expression data sets of atopic dermatitis nonlesional skin. 611 differentially expressed genes were obtained with the threshold of fold change (FC) > 1 and *P* value < 0.05, and the expression value of DEGs among each sample was shown in Figure 3(a). Apart from four samples (GSM815429, GSM815444, GSM815427, and GSM815433), the other samples are well classified. The most significantly enriched BP term and KEGG pathway were “leukocyte migration and PPAR signaling pathway respectively (Figures 3(b) and 3(c)). Furthermore, the GO terms “organic hydroxy compound metabolic process,” “fatty acid metabolic process,” and chemokine signaling pathway were enriched as well.

### 3.2. Specific and Common Characteristics in Psoriasis and Atopic Dermatitis

The specific and shared genes of psoriasis and atopic dermatitis data sets were analyzed. As shown in Figure 4(a), the numbers of DEGs only in psoriasis, atopic dermatitis, and intersection of psoriasis and atopic dermatitis data sets were 498, 377, and 234, respectively. In the meanwhile, the PPI network of 498 DEGs only in psoriasis was analyzed by STRING online software with above-mentioned method (Figure 5). To explore the unique enrichment pathways of psoriasis, GO and KEGG analyses of 498 DEGs were performed. The most significantly enriched BP terms and KEGG pathways were “cornification,” “skin development,” “epidermis development,” and “cytokine-cytokine receptor interaction,” respectively (Figures 4(b) and 4(c)). Furthermore, the GO terms “tissue development,” “response to external biotic stimulus,” “cellular response to cytokine stimulus,” “keratinization,” “neutrophil chemotaxis,” and “cytokine-mediated signaling pathway” were enriched as well.

Similarly, the PPI network of 377 DEGs only in atopic dermatitis was analyzed by STRING online software with abovementioned method (Figure 6). To explore the unique enrichment pathways of atopic dermatitis, GO and KEGG analyses of 377 DEGs were performed. The most significantly enriched BP terms and KEGG pathways were “carboxylic acid metabolic process,” “organic acid metabolic process,” “lipid metabolic process,” “monocarboxylic acid metabolic process,” and PPAR signaling pathway, respectively (Figures 7(a) and 7(b)). Furthermore, the GO terms “fatty acid metabolic process,” “cellular lipid metabolic process,” “lipid biosynthetic process,” and “carboxylic acid catabolic process” were enriched as well.

The article "Exploration of the Potential Mechanism of the Common Differentially Expressed Genes in Psoriasis and Atopic Dermatitis" was published in 2022. Journal: Biomed Res Int.

CXCL8, STAT1, MMP9, and PTPRC were highly expressed in both disease model samples compared with normal samples. Then, we also gained their scores of T cell inflammation in psoriasis and atopic dermatitis data sets, respectively. STAT1 has the highest score of T cell inflammation in both disease (Figures 4(d) and 7(c)).

The expression profile of shared genes among each psoriasis sample was shown in Figure 8(a). Apart from two samples (GSM372333 and GSM372352), the other samples are well classified and the expression pattern diverse among lesional and nonlesional skin samples. Meanwhile, the PPI network of 234 shared DEGs was analyzed by STRING online software with above-mentioned method and shown by Cytoscape software (Figure 8(b)). In this network, the top 20 hub genes were extracted and shown in Table 2. Furthermore, two significant modules of protein-protein network were filtered by using Cytoscape MCODE method, and results were shown in Figure 8(c) (containing 25 nodes and 293 edges) and Figure 8(d) (containing 21 nodes and 195 edges).

We then asked in which pathways these shared DEGs are enriched. To answer this question, we conducted GO and KEGG pathway analysis by ClueGO in Cytoscape, and the results were shown in Figure 9. The enriched BP pathways contain “positive regulation of interleukin-12 production,” “positive regulation of antigen receptor-mediated signaling pathway,” et al. (Figure 9(a)); the enriched CC pathways contain “chromosome,” “centromeric region,” et al. (Figure 9(b)); the enriched MF pathways contain “serine type endopeptidase activity” (Figure 9(c)); the enriched KEGG pathways contain “TNF signaling pathway,” “chemokine signaling pathway,” “IL-17 signaling pathway,” “PPAR signaling pathway,” et al. (Figure 9(d)).

### 3.3. Validation of Common Characteristics in Psoriasis and Atopic Dermatitis

To validate the common characteristics in psoriasis and atopic dermatitis, we tested the expression of above differential genes in mouse model samples. We analyzed gene expression from mouse model of psoriasis and atopic dermatitis by RT-qPCR. As shown in Figures 10(a) and 10(b), CXCL8, STAT1, MMP9 were highly expressed in both disease model samples compared with normal samples. While the expression level of PTPRC was similar between the disease group and the control group. Furthermore, the expression levels of different expressed genes were also detected by Western blot. As shown in Figures 10(c) and 10(d), the psoriasis and atopic dermatitis samples also have high abundances of protein for CXCL8, STAT1, and MMP9 compared with normal samples.

The article "Exploration of the Potential Mechanism of the Common Differentially Expressed Genes in Psoriasis and Atopic Dermatitis" was published in 2022. Journal: Biomed Res Int.

## 4. Discussion

The shared characteristic of two common chronic skin diseases, psoriasis and atopic dermatitis, is extremely vital and helpful for the study of similar pathogenesis, diagnosis, and therapy [25] because of the same disease spectrum [24, 26, 27]. Psoriasis is a chronic inflammatory disease with periodic continuous inflammation and relief, uncontrolled proliferation, and impaired differentiation of keratinocytes [1–3]. Meanwhile, atopic dermatitis (AD) is a chronic inflammatory skin disease related to symptoms such as pruritus, sleep disturbance, depression, and anxiety [14–18]. The DEGs of the two diseases can be used to predict the PPI network and then identify the key hub genes. Betweenness centrality represented the importance of individual node (gene) in the analysis of predicted PPI networks. Simply, the Betweenness of a node stands for the number of shortest paths through the node between all pairs of nodes. Betweenness is a good description of the traffic that a node in a network may need to carry. The greater the Betweenness of a node, the more data packets flow through it, which means that it is more meaningful for the network. The Betweenness of the central node is often very large. Accordingly, the top 20 hub genes in the protein-protein interaction networks of psoriasis and atopic dermatitis have the higher values of Betweenness centrality than the other genes.

Furthermore, there are some specific terms in the psoriasis and atopic dermatitis, respectively. For example, GO terms “tissue development,” “response to external biotic stimulus,” “cellular response to cytokine stimulus,” and “cytokine-mediated signaling pathway” were enriched in the psoriasis data sets. Besides, “keratinization” and “neutrophil chemotaxis” reflect the characteristics of psoriasis; “viral protein interaction with cytokine and cytokine receptor” is also considered as type 1 inflammation. As for the atopic dermatitis data sets, the most significantly enriched BP terms and KEGG pathways were “carboxylic acid metabolic process,” “organic acid metabolic process,” “lipid metabolic process,” and “monocarboxylic acid metabolic process,” which are considered to be related to skin barrier, and “PPAR signaling pathway”, which is related to JAK-STAT, one of the core pathways of atopic dermatitis, respectively.

The article "Exploration of the Potential Mechanism of the Common Differentially Expressed Genes in Psoriasis and Atopic Dermatitis" was published in 2022. Journal: Biomed Res Int.

Besides, the four genes were selected for the validation of their differential expression levels, including CXCL8, STAT1, PTPRC, and MMP9. According to the previous report, abnormal signal transduction in CXCL8-CXCR/2 axis may cause inflammatory diseases including psoriasis and inflammatory bowel diseases [34] which suggests CXCL8 maybe a potential therapeutic target for psoriasis. In addition, CXCL8, STAT1, and MMP9 were upregulated in both psoriasis and atopic dermatitis disease model samples vs. normal samples by the Western blot analyses.

## 5. Conclusion

We brought forth the conclusion that CXCL8, STAT1, and MMP9 may essentially implicate in disease of psoriasis and atopic dermatitis as the potential therapeutic targets.

## Figures and Tables

**Figure 1:** Technical method schematic diagram with the selected data sets in this study.

**Figure 2:** Differential analysis of 33 expression data sets of psoriasis lesional skin and 28 expression data sets of psoriasis nonlesional skin. (a) The heat map of differentially expressed genes from 61 samples. (b) Bubble chart of the top 10 GO-BP (biological process) terms ranked in the gene ratio. (c) Bubble chart of the top 10 KEGG pathways ranked in the gene ratio.

**Figure 3:** Differential analysis of 13 expression data sets of atopic dermatitis lesional skin and 12 expression data sets of atopic dermatitis in nonlesional skin. (a) The heat map of differentially expressed genes from 25 samples. (b) Bubble chart of the top 10 GO-BP (biological process) terms ranked in the gene ratio. (c) Bubble chart of the top 6 KEGG pathways ranked in the gene ratio.

**Figure 4:** Analysis of DEGs only in GSE14905 (psoriasis) data sets. (a) Venn diagram of DEGs in psoriasis (red color) and atopic dermatitis (blue color). (b) Bubble plot of the top 15 GO-BP terms ranked in the gene ratio. (c) Bubble plot of the top 15 KEGG pathways ranked in the gene ratio. (d) T cell inflammation score from GSE14905 (psoriasis) data sets.

**Figure 5:** Predicted protein-protein network of 498 DEGs only in GSE14905 (psoriasis) data sets shown by Cytoscape.

**Figure 6:** Predicted protein-protein network of 377 DEGs only in GSE32924 (atopic dermatitis) data sets shown by Cytoscape.

**Figure 7:** Analysis of DEGs only in GSE32924 (atopic dermatitis) data sets. (a) Bubble plot of the top 15 GO-BP terms ranked in the gene ratio. (b) Bubble plot of the top 15 KEGG pathways ranked in the gene ratio. (c) T cell inflammation score from GSE32924 (atopic dermatitis) data sets.

**Figure 8:** Analysis of DEGs shared in GSE14905 (psoriasis) and GSE32924 (atopic dermatitis) data sets. (a) Heat map of 234 overlapped DEGs in psoriasis. (b) Predicted protein-protein network of 234 overlapped DEGs shown by Cytoscape. The upregulated expressed genes were presented in red circle, whereas the downregulated genes were presented in blue circle. The larger the diameter of the circle is, the higher the degree score is. (c, d) Two modules derived from the protein-protein network in the figure.

The article "Exploration of the Potential Mechanism of the Common Differentially Expressed Genes in Psoriasis and Atopic Dermatitis" was published in 2022. Journal: Biomed Res Int.

**Figure 9:** Enrichment analysis of 234 overlapped DEGs shared in GSE14905 (psoriasis) and GSE32924 (atopic dermatitis) data sets. (a–c) GO enrichment analyses of 234 overlapped DEGs in GO-BP, GO-CC, and GO-MF. (d) KEGG enrichment analyses of 234 overlapped DEGs.

**Figure 10:** The validation of CXCL8, STAT1, PTPRC, and MMP9 in mouse model samples of psoriasis and atopic dermatitis. (a, b) The relative expression of mRNAs in the normal group and the model group of psoriasis (a) and atopic dermatitis (b). (c, d) The abundances of protein CXCL8, STAT1, p-STAT1, PTPRC, MMP9, and control *β*-actin in psoriasis (c, e) and atopic dermatitis (d, f) were determined by Western blot analysis.

**Table 1:** Stem-loop RT and RT-quantitative polymerase chain reaction primer sequences.

Gene	Sequence (5′→3′)
CXCL8 (F)	TGGCAGCCTTCCTGATTT
CXCL8 (R)	AACTTCTCCACAACCCTC
STAT1(F)	CGGAGACAGCCCAGTAAG
STAT1(R)	TGGTCGCAAACGAGACAT
PTPRC(F)	CCACCAGGGACTGACAAG
PTPRC(R)	TTGGGCACGAAGGTTGTC
MMP9(F)	CCCACTTACTATGGAAACTCAA
MMP9(R)	TCAAAGATGAACGGGAACA
Actin(F)	AACAGTCCGCCTAGAAGCAC
Actin(R)	CGTTGACATCCGTAAAGACC

**Table 2:** The top 20 hub genes in the protein-protein interaction network of 234 overlapped DEGs.

Name	Degree	Betweenness centrality	Closeness centrality	Clustering coefficient	Stress	Average shortest path length
CXCL8	46	0.133	0.482	0.204	25680	2.073
STAT1	42	0.085	0.449	0.353	17904	2.225
PTPRC	40	0.116	0.467	0.259	21216	2.14
MMP9	36	0.131	0.466	0.195	26978	2.146
CCL2	35	0.098	0.452	0.291	19580	2.213
CCL5	35	0.027	0.421	0.343	8636	2.376
MKI67	30	0.067	0.392	0.671	13962	2.551
CCNB1	29	0.029	0.389	0.727	8476	2.567
CCR7	28	0.016	0.411	0.378	5186	2.433
CDC20	28	0.014	0.35	0.757	2808	2.854
CDK1	28	0.018	0.361	0.757	3928	2.77
KIAA0101	27	0.031	0.391	0.783	8688	2.556
CXCL1	27	0.018	0.416	0.362	4458	2.404
MX1	27	0.011	0.394	0.624	4112	2.539
IRF1	26	0.011	0.389	0.572	3632	2.573
IRF7	26	0.008	0.386	0.625	3208	2.59
TPX2	26	0.001	0.325	0.871	330	3.073
DLGAP5	26	0.002	0.333	0.88	1026	3
AURKA	26	0.002	0.333	0.88	1026	3
CCNB2	26	0.005	0.341	0.874	1674	2.933

## Data Availability

The data used to support the findings of this study are available from the corresponding author upon request.
